The article "Comparative Pharmacokinetics of Seven Major Compounds in Normal and Atherosclerosis Mice after Oral Administration of Simiao Yong'an Decoction" was published in 2022. Journal: Evid Based Complement Alternat Med.

# Comparative Pharmacokinetics of Seven Major Compounds in Normal and Atherosclerosis Mice after Oral Administration of Simiao Yong'an Decoction

**DOI:** 10.1155/2022/4604601

**Published:** 2022-04-28

**Authors:** Ke-han Sun, Man-fang Yang, Xin-rui Xu, Yang Li, Zhao Gao, Qing-yue Zhang, Hui Li, Shu-qi Wang, Li-xia Lou, Ai-ming Wu, Qiu-shuo Jin, Sheng-xian Wu, Bo Nie

**Affiliations:** ^1^Key Laboratory of Chinese Internal Medicine of Ministry of Education and Beijing, Dongzhimen Hospital, Beijing University of Chinese Medicine, Beijing 100700, China; ^2^School of Chinese Materia Medica, Beijing University of Chinese Medicine, Beijing 100029, China; ^3^Zibo Hospital of Traditional Chinese Medicine, Zibo 255399, Shandong, China

## Abstract

Simiao Yong'an decoction (SMYAD), a classic traditional Chinese medicine formula, has been used to treat atherosclerosis (AS) in clinical in China, but its therapeutic mechanism and pharmacodynamic material basis are not clear. In this study, the AS model was caused by a high-fat diet and perivascular carotid collar placement (PCCP), and SMYAD was orally administered to the model and normal mice. A rapid, sensitive, selective, and reliable method using ultrahigh-performance liquid chromatography (UHPLC) system combined with a Q Exactive HF-X mass spectrometer (UHPLC-Q Exactive HF-X MS) was established and validated for the simultaneous determination of seven compounds, including harpagide, chlorogenic acid, swertiamarin, sweroside, angoroside C, liquiritin, and isoliquiritigenin in the plasma of normal and AS mice. The specificity, linearity, precision, accuracy, recovery, and stability of the method were all within the acceptable criteria. The results showed that some pharmacokinetic behaviors of harpagide, chlorogenic acid, and isoliquiritigenin were significantly different among the two groups of mice. The specific parameter changes were harpagide (AUC_0–*t*_ and AUC_0–∞_ were 11075.09 ± 2132.38 and 16221.95 ± 5622.42 ng·mL^−1^·h, respectively; CLz/F was 2.45 ± 0.87 L/h/mg), chlorogenic acid (*t*_*1/2*_ was 21.59 ± 9.16 h; AUC_0–∞_ was 2637.51 ± 322.54 ng·mL^−1^·h; CLz/F was 13.49 ± 1.81 L/h/mg) and isoliquiritigenin (AUC_0–*t*_ and AUC_0–∞_ were 502.25 ± 165.65 and 653.68 ± 251.34 ng·mL^−1^·h, respectively; CLz/F was 62.16 ± 23.35 L/h/mg) were altered under the pathological status of AS. These differences might be partly ascribed to the changes in gastrointestinal microbiota, nonspecific drug transporters, and cytochrome P450 activity under the AS state, providing research ideas and experimental basis for pharmacological effects and pharmacodynamic material basis.

## 1. Introduction

Atherosclerosis (AS) is the significant pathological basis of cardiovascular and cerebrovascular diseases, which may cause stroke, coronary atherosclerotic heart disease, and myocardial infarction [1]. The pathogenesis of AS is complex and involves various factors, such as endothelial dysfunction, lipid deposition, smooth muscle cell proliferation, oxidative stress, cell apoptosis, and systemic and local inflammation [2]. According to the guideline, lipid-lowering drugs are the first-line drugs for the secondary prevention of coronary heart disease, and statins are the most widely used lipid-lowering drugs in clinical practice [3]. Statins have a significant effect on reducing blood lipid, but there are also adverse reactions, such as muscle symptoms and diabetes in long-term use [4]. Traditional Chinese medicine (TCM) contains a variety of active ingredients, which has good effects on the treatment and prevention of AS in clinical in China [5].

The article "Comparative Pharmacokinetics of Seven Major Compounds in Normal and Atherosclerosis Mice after Oral Administration of Simiao Yong'an Decoction" was published in 2022. Journal: Evid Based Complement Alternat Med.

Simiao Yong'an decoction (SMYAD) is a traditional Chinese medicine formula, which consists of *Lonicera japonica* Thunb. (JYH), *Scrophularia ningpoensis* Hems. (XS), *Angelica sinensis* (Oliv.) Diels (DG), and *Glycyrrhiza uralensis* Fisch. (GC). SMYAD was used to treat gangrene in ancient times according to the traditional Chinese medicine classics. In recent years, this prescription has had a remarkable clinical effect in the treatment of atherosclerosis. It has been confirmed by pharmacological research that SMYAD can affect the migration of smooth muscle cells, inhibit the angiogenesis in plaques, and inhibit the release of inflammatory factors, antioxidative stress, but its pharmacodynamic material basis is indistinct [6, 7]. Previous studies [8, 9] have shown that SMYAD contains many kinds of compounds, such as iridoids, flavonoids, organic acids, and phenylpropanoids. Some of these components have anti-AS-related activities. Harpagide has an effect on facilitating cell migration into the inflamed tissue and promoting the anti-inflammatory activity of the resident macrophages [10]. Chlorogenic acid could protect the ApoE^−/−^ mice against AS through accelerating the cholesterol efflux from macrophages [11]. Swertiamarin has been reported to have high antiatherogenic and cholesterol-lowering potential and can inhibit HMG-Co-A reductase [12]. Sweroside, angoroside C, and liquiritin can take many pharmacological roles, including anti-inflammatory, antioxidation, and cardiovascular protection [13–15]. Isoliquiritigenin could attenuate AS in ApoE^−/−^ mice and inhibit the proliferation of human arterial smooth muscle cell [16, 17]. Since plasma component concentrations and exposure times could well reflect the close relationship between the drug and its pharmacokinetic effect, it is important to interpret the blood components and pharmacokinetic changes for explaining prescription pharmacodynamic substances. Liu et al. investigated the pharmacokinetic characteristics following oral administration of extracts of SMYAD and its single and combined TCMs to rats [18]. However, the data on the pharmacokinetics of SMYAD are limited to normal physiological conditions, and its multicomponent pharmacokinetic investigation in disease conditions has been rarely conducted.

The article "Comparative Pharmacokinetics of Seven Major Compounds in Normal and Atherosclerosis Mice after Oral Administration of Simiao Yong'an Decoction" was published in 2022. Journal: Evid Based Complement Alternat Med.

The ultrahigh-performance liquid chromatography (UHPLC) system combined with a Q Exactive HF-X mass spectrometer can provide high resolution in a short analysis time, allowing the simultaneous detection and quantification of a large number of compounds [19]. Therefore, we developed an analysis method for the simultaneous determination of harpagide, chlorogenic acid, swertiamarin, sweroside, angoroside C, liquiritin, and isoliquiritigenin in normal mice and ApoE^−/−^ mice with a high-fat diet and perivascular carotid collar placement (PCCP)-induced AS using UHPLC-Q Exactive HF-X MS and conducted pharmacokinetic studies in normal and disease conditions. The results will discover the material basis of SMYAD for treating AS to support further drug development, and the pharmacokinetic differences between normal and model mice could provide a reference for the pharmacological mechanism.

## 2. Materials and Methods

### 2.1. Reagents, Chemicals, and Materials

Linarin (internal standard, IS), harpagide, chlorogenic acid, swertiamarin, sweroside, angoroside C, liquiritin, and isoliquiritigenin (purity ≥98%) were purchased from Shanghai Yuanye Bio-Technology Co., Ltd. (Shanghai, China). Methanol (HPLC grade) was purchased from Fisher Scientific (USA). Formic acid (MS grade) was purchased from ANPEL Laboratory Technologies Co., Ltd. (Shanghai, China). The distilled water was purchased from A.S. Watson Group Ltd. (Beijing, China).

*Lonicera japonica* Thunb. (JYH), *Scrophularia ningpoensis* Hems. (XS), *Angelica sinensis* (Oliv.) Diels (DG), and *Glycyrrhiza uralensis* Fisch. (GC) were purchased from the pharmacy of Dongzhimen Hospital of Beijing University of Traditional Chinese Medicine (Beijing, China).

### 2.2. Preparation of SMYAD

Pieces of JYH, XS, DG, and GC were weighed according to the proportion of 3 : 3 : 2 : 1 with appropriate amounts. The mixed pieces were crushed and decocted two times (60 mins first time and 30 mins second time) with water (1 : 10 w/v first time and 1 : 8 w/v second time) after being soaked. The decoctions were then combined and condensed to a concentration of 2 g/mL.

### 2.3. Animal Experiment

Male C57BL/6J mice and ApoE^−/−^ mice on a C57BL/6 background (7 weeks old, 18–22 g) were purchased from Beijing Vital River Laboratory Animal Technology Co., Ltd. (Beijing, China, Certificate No.: SCXK (Jing) 2016-0006). All the mice were kept in an SPF animal house (Dongzhimen Hospital Affiliated to Beijing University of Chinese Medicine, Certificate No.: SYXK (Jing) 2015-0001) with food and water freely available, 12 h light/dark, and environmental conditions of 22°C–24°C, 50% relative humidity. All protocols of animal experiments were performed in accordance with the National Guidelines for Laboratory Animal Welfare and were approved by the Animal Ethics Committee of Beijing University of Chinese Medicine (NO. BUCM-4-2015071701-3001). High-fat feeding (containing 15% fat and 0.25% cholesterol) was provided by Beijing HFK bioscience CO., LTD. (Beijing, China, Certificate No.: SCXK (Jing) 2014-0018).

The article "Comparative Pharmacokinetics of Seven Major Compounds in Normal and Atherosclerosis Mice after Oral Administration of Simiao Yong'an Decoction" was published in 2022. Journal: Evid Based Complement Alternat Med.

The AS model was established by a high-fat diet and perivascular carotid collar placement (PCCP) surgery in the ApoE^−/−^ mice. After a 7-day adaptive feeding, the mice were given a high-fat diet for 2 weeks; before anesthesia, all ApoE^−/−^ mice were fasted for 12 hours. During the surgery, the right common carotid artery was exposed, and a silicone cannula (length: 2.5 mm, inner diameter: 0.3 mm) was fixed around the carotid artery (external diameter: about 0.5 mm). Penicillin was injected intraperitoneally for 3 days after surgery to prevent infection. High-fat diet continued for 8 weeks after surgery to establish AS model. Biochemical assays and hematoxylin and eosin (HE) staining were used to evaluate whether AS model was successfully established.

The serum concentrations of total cholesterol (TC), triacylglycerols (TG), low-density lipoprotein cholesterol (LDL-C), and high-density lipoprotein cholesterol (HDL-C) were determined by the automatic biochemical analyzer (AU5800, Beckman Coulter Co., Ltd.). The right carotid arteries of the mice were obtained under stereoscopic observation and fixed by 4% paraformaldehyde, and every consecutive section (3 *μ*m thick) throughout the right carotid artery of the mice was stained with HE.

### 2.4. Pharmacokinetic Study

Normal control (NC) and AS mice (30 per group) were employed to investigate the pharmacokinetic properties of harpagide, chlorogenic acid, swertiamarin, sweroside, angoroside C, liquiritin, and isoliquiritigenin after the oral administration of SMYAD. After successful induction of AS model, SMYAD was administered to NC and AS mice by intragastric gavage at the crude drug dose of 35 g/kg/d for seven days. Blood samples were collected from each mouse in heparinized tubes via the postorbital venous plexus veins at 0, 0.25, 0.5, 1, 2, 4, 6, 8, 10, 12, 18, and 24 h after seven days of drug administration. Then blood samples were immediately centrifuged at 3500 rpm at 4°C for 10 min and the plasma was stored at −80°C until use.

The article "Comparative Pharmacokinetics of Seven Major Compounds in Normal and Atherosclerosis Mice after Oral Administration of Simiao Yong'an Decoction" was published in 2022. Journal: Evid Based Complement Alternat Med.

### 2.5. Preparation of Stocks Calibration Standard and Quality Control (QC) Samples

Stock solutions of linarin (internal standard, IS), harpagide, chlorogenic acid, swertiamarin, sweroside, angoroside C, liquiritin, and isoliquiritigenin were dissolved in methanol at the concentration of 100 *μ*g/mL, respectively. Then the mixed stock solution was obtained by 6 *μ*g/mL of harpagide, 8 *μ*g/mL of chlorogenic acid, 48 *μ*g/mL of swertiamarin, 10 *μ*g/mL of sweroside, 2 *μ*g/mL of angoroside C, liquiritin, and isoliquiritigenin. The IS working solution was diluted with the methanol to a final concentration of 400 ng/mL.

Standard calibration curves were constructed by spiking 100 *μ*L of blank mouse plasma with 25 *μ*L of the standard working solutions and 25 *μ*L of the IS working solution, yielding final plasma concentrations in the range of 2–1500 ng/mL for harpagide, 1–2000 ng/mL for chlorogenic acid, 5–12000 ng/mL for swertiamarin, 5–2500 ng/mL for sweroside, 5–500 ng/mL for angoroside C and liquiritin, and 2–500 ng/mL for isoliquiritigenin.

Quality control (QC) samples at three concentration levels (38.4, 240, and 600 ng/mL for harpagide; 51.2, 320, and 800 ng/mL for chlorogenic acid; 307.2, 1920, and 4800 ng/mL for swertiamarin; 64, 400, and 1000 ng/mL for sweroside; 12.8, 80, and 200 ng/mL for angoroside C, liquiritin, and isoliquiritigenin) were prepared by the same operation described above. All solutions were stored at 4°C.

### 2.6. Preparation of Plasma Samples

Each plasma sample (100 *μ*L) was mixed with a threefold volume of methanol and 25 *μ*L IS in a 1.5 mL EP tube. Then the mixture was vortexed for 100 seconds and centrifuged at 12,000 rpm for 10 min at 4°C. The supernatant was transferred to another EP tube and evaporated to dryness under a nitrogen vacuum. The residue was reconstituted with 100 *μ*L of 50% methanol and centrifuged at 15,000 rpm for 15 min. Then the supernatant was transferred to sample vials for the LC-MS analysis.

### 2.7. Instruments and Experimental Conditions

A Vanquish UHPLC™ system (Thermo Fisher Scientific Inc., USA) was used for the analysis. Samples were separated on an Atlantis T3 column (4.6 mm × 150 mm, 3 *μ*m; Waters, USA). The column temperature was 40°C. The mobile phase, at 0.4 mL/min, consisted of water containing 0.1% formic acid (v/v, A) and methanol (B). The quantitative analysis gradient program was as follows: 0-1 min, 0 B; 1–6 min, 0–100% B; 6–12 min, 100% B; 12–12.1 min, 100%-0 B; 12.1–15 min, 0 B. The injection volume was 5 *μ*L.

The article "Comparative Pharmacokinetics of Seven Major Compounds in Normal and Atherosclerosis Mice after Oral Administration of Simiao Yong'an Decoction" was published in 2022. Journal: Evid Based Complement Alternat Med.

The mass spectrometer Q Exactive HF-X (Thermo Fisher Scientific Inc., USA) system was connected to the UHPLC system via heated electrospray ionization (HESI) and controlled by Xcalibur 4.2 software (Thermo Fisher) that was used for data collection and analysis. The mass spectrometer was operated in a negative ionization mode. The MS parameters were set as follows: probe heater temperature, 350°C; capillary temperature: 320°C; sheath gas (N2) flow rate: 30 arbs; auxiliary gas (N2) flow rate: 10 arbs; spray voltage: 3.2 kV (negative); S-Lens RF level: 55 V; scan mode: full MS (resolution 12000); scan range: m/z 150–1500. The most abundant ions in the spectra were selected for sensitive quantitation ([M-H]^−^of chlorogenic acid, angoroside C, liquiritin, isoliquiritigenin, and IS, [M + COOH]^−^ of harpagide, swertiamarin, and sweroside). The m/z of harpagide was 409.13405, chlorogenic acid was 353.08671, swertiamarin was 419.11840, sweroside was 403.12349, angoroside C was 783.27061, liquiritin was 417.11801, isoliquiritigenin was 255.06519, and IS was 591.17083. The structures and mass spectrum of seven analytes and IS are shown in Figure 1.

### 2.8. Data Analysis

The pharmacokinetic parameters, including maximum plasma concentration (*C*_max_), time corresponding to *C*_max_ (*T*_max_), terminal elimination half-life (*T*_1/2_), area under plasma concentration-time curve (AUC_0–*t*_) and area under the plasma concentration-time curve from 0 to infinity time (AUC_0–∞_), apparent volume of distribution (Vz/F) and clearance (CLz/F), were calculated using the noncompartment model in DAS 2.0 software package (Shanghai, China). GraphPad prism 6.02 (GraphPad Software, USA) was used in the statistical analysis. All values are expressed as mean ± standard error. For the pharmacokinetic parameter values of the NC and AS groups, Student's *t*-test was employed for data comparisons. *P* values <0.05 were considered statistically significant.

## 3. Results and Discussion

### 3.1. ApoE^−/−^ Mice as Model Were Successfully Established

Serum biochemical parameters of mice including TC, TG, LDL-C, and HDL-C were determined (see Table 1). Compared to the normal group, TC and LDL-C levels were significantly increased in the AS model group (*P* < 0.01), and there were no significant differences in TG and HDL-C levels between the two groups.

HE staining (see Figure 2) showed that the NC group had intact carotid artery structure and no obvious AS plaque formation. Compared with the NC group, the AS group showed AS plaque protruding to the lumen, the vascular lumen was significantly narrowed, foam cells were piled up in the intima, the smooth muscle was disordered and migrated to the intima, and AS plaque was obviously formed. The above results indicated that the AS model was successfully established.

The article "Comparative Pharmacokinetics of Seven Major Compounds in Normal and Atherosclerosis Mice after Oral Administration of Simiao Yong'an Decoction" was published in 2022. Journal: Evid Based Complement Alternat Med.

### 3.2. Method Validation

#### 3.2.1. Specificity

The selectivity was evaluated by comparing the typical chromatograms of blank plasma (in Figure 3(a)), the blank plasma spiked with the seven target analytes and IS (in Figure 3(b)), and the plasma after oral administration of SMYAD (in Figure 3(c)). There was no endogenous interference in the full scan mode for each of the analytes in all samples, indicating the good specificity of the analysis method.

#### 3.2.2. Linearity and Lower Limit of Quantification (LLOQ)

The calibration curves for the seven components were established by plotting the peak area ratios of each analyte to the IS against plasma concentrations using the least-square linear regression with a weighted (1/*x*) factor. The limit of detection (LOD) was determined for a signal-to-noise(S/N) ratio of more than 3. The lower limit of quantification (LLOQ) was determined as the lowest concentration on the calibration curve (S/N > 10). As shown in Table 2, the standard curves of the seven target analytes had good linearity with correlation coefficients more than 0.9969. The lowest LLOQ was 1.0 ng/mL.

#### 3.2.3. Recovery and Matrix Effect

The extraction recoveries and matrix effects of the seven compounds were evaluated by determining the QC samples at three concentration levels with five replicates. The recovery of six analytes was measured by comparing the peak areas obtained from the extracted QC samples with those obtained from mixed standards spiked into postextracted blank plasma. The matrix effect was expressed as comparing the peak response of the analytes in plasma samples with those of the pure standards prepared in methanol. The extraction recoveries were in the acceptable range from 90.17% to 111.33%. Regarding the matrix effects, all ratios were between 89.23% and 112.72%, suggesting that there were no endogenous substances and interference for the ionization of the analytes in the coeluting matrix (see Table 3).

#### 3.2.4. Precision and Accuracy

Precision and accuracy were evaluated as five replicate QC samples at LLOQ, low, middle, and high four concentration levels. Intraday precision and accuracy were analyzed during the same day while interday precision and accuracy were investigated on three successive days. Precision (relative standard deviation, RSD) and accuracy (RE) for intra- and interday values were below 15% and within ±15% for the seven compounds (see Table 4), respectively. The results indicated that the intra- and interday precision (RSD%) of these analytes were in the range of 9.39% to 10.5%, respectively, while the corresponding REs ranged from −9.73% to 13.69%, respectively. These results suggested that this method had an acceptable precision and accuracy.

The article "Comparative Pharmacokinetics of Seven Major Compounds in Normal and Atherosclerosis Mice after Oral Administration of Simiao Yong'an Decoction" was published in 2022. Journal: Evid Based Complement Alternat Med.

#### 3.2.5. Stability

Stability was evaluated as five replicate QC samples at two concentration levels (see Table 5). The extracted samples were stable under the testing conditions including autosampler temperature (4°C) for 24 h, room temperature (20°C) for 24 h, three freeze-thaw cycles, and long-term cold storage (−20°C for 30 days) with RE% values of −13.11% to 11.89%, indicating that all active ingredients were stable during the analysis.

### 3.3. Pharmacokinetic Study

The validated method was successfully utilized to examine the concentrations of harpagide, chlorogenic acid, swertiamarin, sweroside, angoroside C, liquiritin, and isoliquiritigenin in NC and AS mice plasma. The mean blood concentration-time curves of seven active components after oral administration of SMYAD (35 g/kg/day) in NC and AS mice are illustrated in Figure 4, and the main pharmacokinetic parameters are listed in Table 6.

The results suggested that active components harpagide, chlorogenic acid, swertiamarin, sweroside, angoroside C, liquiritin, and isoliquiritigenin were quickly absorbed in NC and AS mice after oral administration of SMYAD showing good pharmacokinetic parameters, which was consistent with previous reports [14, 15, 20–24].

Compared with the normal mice, the trends of plasma concentration-time curves of the seven ingredients were changed in AS mice. In terms of pharmacokinetic parameters, the absorption of some active ingredients in AS mice was altered. Specifically, the AUC_0–*t*_ of harpagide (11075.09 ± 2132.38 ng·mL^−1^·h, *P* < 0.01), the AUC_0–∞_ of hapagide (16221.95 ± 5622.42 ng·mL^−1^·h, *P* < 0.05), and the chlorogenic acid (2637.51 ± 322.54 ng·mL^−1^·h, *P* < 0.01) in the AS group significantly increased compared with the normal group, indicating that harpagide and chlorogenic acid exhibited high absorption in AS status. For swertiamarin, sweroside, and angoroside C, the increased tendencies of AUC_0–t_ and AUC_0–∞_ value were also observed, but no significant difference was discovered. However, significant reduction of AUC_0–t_ (502.25 ± 165.65 ng·mL^−1^·h, *P* < 0.01) and the AUC_0–∞_ (653.68 ± 251.34 ng·mL^−1^·h, *P* < 0.05) for isoliquiritigenin in the AS group were discovered, indicating that the bioavailability of isoliquiritigenin was remarkably reduced in the AS group. For liquiritin, the decreased tendencies of AUC_0–t_ and AUC_0–∞_ were also observed, but no significant difference was discovered. Furthermore, a longer *T*_1/2_ for chlorogenic acid (21.59 ± 9.16 h, *P* < 0.05) wase observed in the AS group compared with the NC group, whereas no significant change in *T*_1/2_ was observed for other compounds between the two groups. And the obvious lower CLz/F (*P* < 0.01) of harpagide and chlorogenic acid compared with NC group were observed, which means the metabolic rate of the two compounds slow down under pathological conditions. However, a significant increase in CLz/F (*P* < 0.05) of isoliquiritigenin was observed in the AS group. The results indicated that the oral administration of SMYAD could lead to slower elimination of chlorogenic acid and harpagide, but the elimination of isoglycyrrhizin was accelerated in AS mice. In addition, The Vz/F value of these compounds in both normal and model was large, indicating that the active compounds in SMYAD were possibly bound to tissue proteins, mainly distributed in tissue and intracellular fluids.

The article "Comparative Pharmacokinetics of Seven Major Compounds in Normal and Atherosclerosis Mice after Oral Administration of Simiao Yong'an Decoction" was published in 2022. Journal: Evid Based Complement Alternat Med.

The pathogenesis of AS is complex, and inflammatory reaction runs through the whole process of plaque rupture and thrombosis, especially unstable plaque rupture [25]. AS is often accompanied by a number of metabolic syndromes such as glycometabolism dysfunction and lipid-metabolism dysfunction. Under the pathological conditions of AS, the absorption, distribution, metabolism, and excretion of the main bioactive components of SMYAD may be affected by complex factors. The possible reasons for pharmacokinetic differences between normal and AS model mice may be addressed by the following explanations. It was reported that the abundance and composition of the gut microbiota were altered in AS patients [26]. The gut microbiota has the genetic mechanisms necessary to produce enzymes that metabolize oral drugs, focusing on two main types of reactions: hydrolysis and reduction. Microbial metabolism converts hydrophilic drugs into hydrophobic compounds, thereby enhancing their absorption in the gut, and the hydrolytic enzyme activities of intestinal flora may decrease in the atherosclerotic disease state [27], while the level of related proinflammatory factors (NF-*κ*B, TNF-*α*, IL-1*β*, and IL-6) increases in AS [28]. Study [29] has shown that the increase of inflammatory factors will further reduce the expression of some enzymes, and these may be the cause of the slow metabolism of harpagide and chlorogenic acid, the increased absorption for harpagide and chlorogenic acid, and the decreased absorption for isoliquiritigenin in AS model mice. The cause of their absorption changes may also be relative to nonspecific drug transporters, such as P-glycoprotein. Changes in normal and AS status drug transporters can be further studied. Research [30] suggested that marked inhibition of hepatic cytochrome P450 activity in cholesterol-induced atherosclerosis in rabbits and decreased metabolism of harpagide and chlorogenic acid in AS mice may be related to the decrease in CYP450 activity in the disease state. All the above considerations suggested that the anti-AS mechanisms of SMYAD should be based on gut microbiota, drug transporters, and CYP450 activity.

The article "Comparative Pharmacokinetics of Seven Major Compounds in Normal and Atherosclerosis Mice after Oral Administration of Simiao Yong'an Decoction" was published in 2022. Journal: Evid Based Complement Alternat Med.

Harpagide, chlorogenic acid, and isoliquiritigenin have anti-inflammatory, inhibition of oxidative stress, lowering blood lipids, and other pharmacological activities to ameliorate AS. Therefore, it is speculated that these components may be the key active constituents of SMYAD in the treatment of AS. In addition, there was a large difference in mean blood concentration at some time points, and some pharmacokinetic parameters showed the trend of difference between normal and model, but it was not statistically significant, which may be the reason for the small sample size.

## 4. Conclusions

A sensitive, rapid, and reliable UHPLC-Q Exactive HF-X MS analytical method was established and validated for the simultaneous determination and quantification of harpagide, chlorogenic acid, swertiamarin, sweroside, angoroside C, liquiritin, and isoliquiritigenin in the plasma of normal and AS mice. It is the first comparative study of the pharmacokinetics of seven active components of SMYAD in normal and AS mice. The results demonstrated that AUC of harpagide and chlorogenic acid was significantly increased and CLz/F was decreased, meanwhile *t*_*1/2*_ of chlorogenic acid was prolonged, while the AUC of isoliquiritigenin was decreased and its CLz/F was increased. Pharmacokinetic behaviors of swertiamarin, sweroside, angoroside C, and liquiritin were not changed obviously after oral administration of SMYAD in normal and AS model. This study laid the experimental foundation for further elucidating the pharmacodynamic substances of SMYAD against AS, and the difference in pharmacokinetic parameters provided a scientific reference for clarifying the targets of SMYAD *in vivo*.

## Figures and Tables

**Figure 1:** Chemical structures and mass spectrum of the seven compounds and IS.

**Figure 2:** HE-stained carotid artery sections from NC and AS model. (a) NC group; (b) AS group (magnification, ×20).

**Figure 3:** Extracted-ion chromatograms of harpagide, chlorogenic acid, swertiamarin, sweroside, angoroside C liquiritin, isoliquiritigenin, and IS. (a) Blank plasma; (b) blank plasma spiked with the seven target analytes and IS; (c) drug-containing plasma after administration of SMYAD.

**Figure 4:** Mean concentration-time curves of seven compounds in NC and ASmouse plasma after oral administration of SMYAD (mean ± SD, *n* = 5). (a) Harpagide; (b) chlorogenic acid; (c) swertiamarin; (d) sweroside; (e) angoroside C; (f) liquiritin; (g) isoliquiritigenin.

The article "Comparative Pharmacokinetics of Seven Major Compounds in Normal and Atherosclerosis Mice after Oral Administration of Simiao Yong'an Decoction" was published in 2022. Journal: Evid Based Complement Alternat Med.

**Table 1:** Comparison of blood lipids in the normal group and model group (mean ± SD, *n* = 6, mmol/L).

Group	TC	TG	HDL-C	LDL-C
NC	2.42 ± 0.28	1.64 ± 0.33	1.35 ± 0.18	0.35 ± 0.06
AS	29.15 ± 0.78^*∗∗*^	1.35 ± 0.26	1.16 ± 0.10	7.39 ± 0.69^*∗∗*^

Compared with the NC group, ^*∗*^*P* < 0.05, ^*∗∗*^*P* < 0.01.

**Table 2:** Liner range, regression equation, and correlation coefficient for seven compounds.

Compounds	Liner range (ng/ml)	Regression equation	Correlation coefficient (*r*^2^)	LOD (ng/mL)	LLOQ (ng/mL)
Harpagide	2∼1500	*y* = 0.0021x − 0.0015	0.9982	1	2
Chlorogenic acid	1∼2000	*y* = 0.0020x + 0.0131	0.9978	0.5	1
Swertiamarin	5∼12000	*y* = 0.0040x − 0.0118	0.9980	2.5	5
Sweroside	5∼2500	*y* = 0.0056x + 0.0241	0.9969	2.5	5
Angoroside C	5∼500	*y* = 0.0027x − 0.0053	0.9981	2.5	5
Liquiritin	5∼500	*y* = 0.0150x + 0.0040	0.9998	2.5	5
Isoliquiritigenin	2∼500	*y* = 0.0297x − 0.0562	0.9968	1	2

**Table 3:** Recovery and the matrix effect of seven target analytes in QC plasma samples (*n* = 5).

Compounds	QC conc. (ng/mL)	Recovery (%)		Matrix effect (%)	
		Mean (%)	RSD (%)	Mean (%)	RSD (%)
Harpagide	600	101.14	6.37	95.40	3.74
	240	110.32	13.18	91.60	11.41
	38.4	96.61	7.33	96.65	3.13

Chlorogenic acid	800	104.87	5.66	112.72	10.05
	320	107.35	13.24	105.99	6.96
	51.2	100.99	5.50	95.46	4.97

Swertiamarin	4800	99.16	2.23	98.75	3.36
	1920	111.33	1.76	92.09	3.75
	307.2	92.68	9.61	92.37	6.59

Sweroside	1000	102.26	4.23	97.44	3.29
	400	109.48	6.11	89.23	2.33
	64	103.26	7.61	94.33	6.33

Angoroside C	200	98.04	4.06	106.36	6.23
	80	108.81	11.18	103.66	4.81
	12.8	90.17	12.76	109.11	11.46

Liquiritin	200	109.31	6.04	102.86	3.65
	80	106.23	6.80	100.54	3.08
	12.8	103.04	13.81	92.59	5.93

Isoliquiritigenin	200	92.80	8.01	108.26	2.50
	80	106.81	10.11	112.06	6.92
	12.8	94.89	7.79	110.64	11.11

**Table 4:** Precision and accuracy of seven target analytes in QC plasma samples (mean ± SD, *n* = 15).

Compounds	QC conc. (ng/ml)	Intraday			Inter-day		
		Calc. conc. (ng/ml)	Precision RSD (%)	Accuracy RE (%)	Calc. conc. (ng/ml)	Precision RSD (%)	Accuracy RE (%)
Harpagide	600	621.92 ± 33.83	5.44	3.65	625.92 ± 44.85	7.17	4.32
	240	216.64 ± 10.24	4.73	−9.73	230.99 ± 18.93	8.19	−3.75
	38.4	40.84 ± 3.07	7.51	6.36	39.58 ± 3.30	8.33	3.07
	2	1.74 ± 0.07	3.75	−13.21	1.88 ± 0.23	11.98	−6.03

Chlorogenic acid	800	816.65 ± 48.51	5.94	2.08	827.94 ± 49.36	5.96	3.49
	320	352.34 ± 12.96	3.68	10.11	337.79 ± 24.01	7.11	5.56
	51.2	53.83 ± 5.05	9.39	5.14	53.31 ± 4.59	8.62	4.12
	1	0.97 ± 0.09	9.20	−3.36	0.97 ± 0.08	8.02	−3.35

Swertiamarin	4800	5457.20 ± 189.52	3.47	13.69	5238.94 ± 266.24	5.08	9.14
	1920	1980.91 ± 65.11	3.29	3.17	2056.51 ± 84.80	4.12	7.11
	307.2	297.15 ± 6.53	2.20	−3.27	304.89 ± 18.84	6.18	−0.75
	5	4.37 ± 0.31	7.09	−12.54	5.30 ± 0.70	13.30	5.96

Sweroside	1000	1084.72 ± 35.82	3.30	8.47	1071.96 ± 52.80	4.93	7.20
	400	396.99 ± 14.08	3.55	−0.75	418.16 ± 24.41	5.84	4.54
	64	63.54 ± 4.14	6.52	−0.73	64.87 ± 5.66	8.73	1.36
	5	5.09 ± 0.43	8.51	1.84	4.77 ± 0.41	8.57	−4.70

Angoroside C	200	190.43 ± 10.30	5.41	−4.79	198.76 ± 15.54	7.82	−0.62
	80	81.37 ± 4.63	5.70	1.71	79.58 ± 8.35	10.50	−0.53
	12.8	12.19 ± 0.81	6.63	−4.80	12.62 ± 1.08	8.59	−1.43
	5	4.51 ± 0.29	6.47	−9.86	4.41 ± 0.36	8.17	−11.80

Liquiritin	200	204.79 ± 5.51	2.69	2.39	190.27 ± 12.20	6.41	−4.86
	80	77.78 ± 1.25	1.60	−2.78	75.51 ± 3.80	5.03	−5.61
	12.8	13.15 ± 0.79	5.99	2.76	13.11 ± 0.96	7.30	2.42
	5	4.89 ± 0.47	9.54	−2.14	4.51 ± 0.44	9.86	−9.85

Isoliquiritigenin	200	218.31 ± 6.58	3.01	9.16	216.37 ± 7.84	3.62	8.19
	80	79.91 ± 3.17	3.97	−0.11	78.55 ± 3.72	4.73	−1.81
	12.8	13.68 ± 0.41	3.02	6.85	13.16 ± 1.01	7.70	2.80
	2	1.97 ± 0.21	10.68	−1.41	1.95 ± 0.25	12.92	−2.64

The article "Comparative Pharmacokinetics of Seven Major Compounds in Normal and Atherosclerosis Mice after Oral Administration of Simiao Yong'an Decoction" was published in 2022. Journal: Evid Based Complement Alternat Med.

**Table 5:** Stability of seven target analytes in QC plasma samples (mean ± SD, *n* = 5).

Compounds	QC (ng/ml)	Postpreparative stability 24 h in the autosampler (4°C)		Short-term stability 24 h in room temperature (20°C)		Freeze-thaw stability 3 freeze-thaw cycles		Long-term stability −20°C for 30 d	
		Calc. conc. (ng/ml)	Accuracy RE (%)	Calc. conc. (ng/ml)	Accuracy RE (%)	Calc. conc. (ng/ml)	Accuracy RE (%)	Calc. conc. (ng/ml)	Accuracy RE (%)
Harpagide	600	575.51 ± 22.16	−4.08	654.47 ± 22.87	9.08	587.47 ± 36.62	−2.09	612.90 ± 22.28	2.15
	38.4	38.35 ± 3.75	−0.13	39.34 ± 1.92	2.45	38.05 ± 4.19	−0.92	40.68 ± 3.21	5.94

Chlorogenic acid	800	833.85 ± 63.43	4.23	816.58 ± 29.60	2.07	863.78 ± 21.49	7.97	847.20 ± 32.63	5.90
	51.2	53.43 ± 3.66	4.35	49.06 ± 4.43	−4.19	56.51 ± 2.77	10.38	51.69 ± 5.02	0.96

Swertiamarin	4800	4968.64 ± 208.19	3.51	5274.04 ± 147.92	9.88	5153.93 ± 132.15	7.37	4835.93 ± 153.29	0.75
	307.2	292.85 ± 19.45	−4.67	279.92 ± 15.61	−8.88	289.21 ± 13.27	−5.86	311.53 ± 14.38	1.41

Sweroside	1000	1035.71 ± 53.35	3.57	1113.06 ± 32.37	11.31	1079.40 ± 37.61	7.94	973.49 ± 29.27	−2.65
	64	60.97 ± 4.81	−4.74	66.44 ± 4.64	3.81	63.90 ± 2.67	−0.16	63.40 ± 2.49	−0.94

Angoroside C	200	185.46 ± 9.39	−7.27	203.84 ± 4.39	1.92	196.52 ± 13.15	−1.74	178.97 ± 6.04	−10.51
	12.8	13.02 ± 1.05	1.70	13.32 ± 1.09	4.09	13.53 ± 0.98	5.68	13.02 ± 1.17	1.73

Liquiritin	200	173.78 ± 5.96	−13.11	189.11 ± 4.81	−5.45	180.23 ± 4.39	−9.88	184.99 ± 6.52	−7.50
	12.8	13.43 ± 0.75	4.90	12.47 ± 0.97	−2.58	12.41 ± 0.76	−3.04	13.40 ± 0.70	4.70

Isoliquiritigenin	200	220.77 ± 9.12	10.39	192.67 ± 7.93	−3.66	223.78 ± 4.10	11.89	177.89 ± 4.50	−11.06
	12.8	13.27 ± 0.64	3.66	13.72 ± 0.54	7.15	13.83 ± 1.09	8.02	13.81 ± 0.76	7.87

The article "Comparative Pharmacokinetics of Seven Major Compounds in Normal and Atherosclerosis Mice after Oral Administration of Simiao Yong'an Decoction" was published in 2022. Journal: Evid Based Complement Alternat Med.

**Table 6:** Main pharmacokinetic parameters of the seven compounds in mouse plasma after oral administration of SMYAD (mean ± SD, *n* = 5).

Compounds	Group	Parameters						
		*t*_*1/2*_ */*h	*t*_max_/h	*C*_max_/ng·mL^−1^	AUC_0–*t*_/ng·mL^−1^·h	AUC_0–∞_/ng·mL^−1^·h	Vz/F (L/mg)	CLz/F (L/h/mg)
Harpagide	NC	8.40 ± 1.80	6.00 ± 2.19	838.40 ± 126.54	6936.17 ± 533.23	7194.33 ± 588.34	32.74 ± 7.64	4.90 ± 0.40
	AS	8.55 ± 3.97	4.00 ± 0.00	939.74 ± 180.83	11075.09 ± 2132.38^*∗∗*^	16221.95 ± 5622.42^*∗*^	24.34 ± 16.57	2.45 ± 0.87^*∗∗*^

Chlorogenic acid	NC	4.51 ± 1.10	1.13 ± 0.88	266.84 ± 72.39	1109.84 ± 418.97	1257.70 ± 424.87	247.01 ± 150.71	30.37 ± 7.58
	AS	21.59 ± 9.16^*∗*^	0.25 ± 0.00	1128.91 ± 969.58	1560.11 ± 476.37	2637.51 ± 322.54^*∗∗*^	302.49 ± 211.89	13.49 ± 1.81^*∗∗*^

Swertiamarin	NC	4.43 ± 2.06	5.00 ± 4.97	1431.10 ± 636.23	5349.68 ± 1183.98	5401.77 ± 1243.88	20.82 ± 11.26	5.82 ± 2.64
	AS	5.74 ± 1.90	0.90 ± 0.64	1335.08 ± 603.03	5542.40 ± 2011.02	7243.79 ± 3391.00	55.16 ± 45.04	5.70 ± 1.93

Sweroside	NC	3.81 ± 0.56	0.40 ± 0.30	1793.48 ± 368.69	6983.11 ± 381.87	7083.75 ± 389.99	16.99 ± 3.78	4.96 ± 0.28
	AS	6.56 ± 2.75	0.90 ± 0.64	1588.23 ± 496.61	7501.27 ± 1799.94	8926.84 ± 2117.67	29.99 ± 14.26	4.29 ± 1.55

Angoroside C	NC	7.40 ± 4.76	0.85 ± 0.62	288.62 ± 123.79	1732.42 ± 882.96	1865.70 ± 1053.21	148.22 ± 76.23	29.75 ± 24.10
	AS	7.33 ± 4.68	2.05 ± 1.19	491.04 ± 238.94	1838.19 ± 298.23	1891.33 ± 226.37	126.00 ± 102.72	18.79 ± 2.39

Liquiritin	NC	16.98 ± 3.43	0.75 ± 0.63	132.03 ± 57.09	606.62 ± 229.46	760.40 ± 333.88	565.81 ± 116.60	58.74 ± 30.94
	AS	13.54 ± 3.57	0.75 ± 0.69	67.62 ± 33.62	407.58 ± 115.29	481.57 ± 137.03	887.57 ± 397.82	67.62 ± 33.62

Isoliquiritigenin	NC	6.65 ± 1.31	1.90 ± 2.13	175.33 ± 49.02	1036.28 ± 144.06	1063.27 ± 144.39	198.37 ± 58.53	33.51 ± 4.41
	AS	6.01 ± 2.32	0.95 ± 0.60	134.59 ± 101.80	502.25 ± 165.65^*∗∗*^	653.68 ± 251.34^*∗*^	658.87 ± 555.51	62.16 ± 23.35^*∗*^

Compared with the NC group, ^*∗*^*P* < 0.05, ^*∗∗*^*P* < 0.01.

## Data Availability

The data used to support the findings of this study are included within the article.
